# Prediction Performance of Deep Learning for Colon Cancer Survival Prediction on SEER Data

This article has been retracted.

**DOI:** 10.1155/2022/1467070

**Published:** 2022-06-16

**Authors:** Surbhi Gupta, S. Kalaivani, Archana Rajasundaram, Gaurav Kumar Ameta, Ahmed Kareem Oleiwi, Betty Nokobi Dugbakie

**Affiliations:** ^1^Model Institute of Engineering & Technology, Jammu, J&K, India; ^2^School of Information Technology and Engineering, Vellore Institute of Technology (VIT), Vellore, Tamil Nadu, India; ^3^Department of Anatomy, Sree Balaji Medical College and Hospital, Chennai, Tamil Nadu, India; ^4^Department of Computer Engineering, Indus Institute of Technology & Engineering, Indus University, Ahmedabad, Gujarat, India; ^5^Department of Computer Technical Engineering, The Islamic University, 54001 Najaf, Iraq; ^6^Department of Chemical Engineering, Kwame Nkrumah University of Science and Technology (KNUST), Ghana

## Abstract

Colon and rectal cancers are the most common kinds of cancer globally. Colon cancer is more prevalent in men than in women. Early detection increases the likelihood of survival, and treatment significantly increases the likelihood of eradicating the disease. The Surveillance, Epidemiology, and End Results (SEER) programme is an excellent source of domestic cancer statistics. SEER includes nearly 30% of the United States population, covering various races and geographic locations. The data are made public via the SEER website when a SEER limited-use data agreement form is submitted and approved. We investigate data from the SEER programme, specifically colon cancer statistics, in this study. Our objective is to create reliable colon cancer survival and conditional survival prediction algorithms. In this study, we have presented an overview of cancer diagnosis methods and the treatments used to cure cancer. This paper presents an analysis of prediction performance of multiple deep learning approaches. The performance of multiple deep learning models is thoroughly examined to discover which algorithm surpasses the others, followed by an investigation of the network's prediction accuracy. The simulation outcomes indicate that automated prediction models can predict colon cancer patient survival. Deep autoencoders displayed the best performance outcomes attaining 97% accuracy and 95% area under curve-receiver operating characteristic (AUC-ROC).

## 1. Introduction

Cancer prediction and diagnosis is a complex subject that has piqued the interest of researchers worldwide due to the disease's high morbidity and mortality [1, 2]. Furthermore, cancer has been regarded as a multifaceted disease with several subtypes. Early diagnosis and prognosis of a cancer type has become a requirement in cancer research since it can aid in patient clinical therapy [3, 4]. Early cancer detection increases the chances of a successful therapy. The two components of cancer early detection are early diagnosis (or downstaging) and screening. Initial diagnosis is concerned with finding problematic patients as soon as possible, whereas screening is concerned with examining healthy persons to detect cancers before symptoms appear. Screening programmes should be implemented only after their efficacy has been demonstrated, when resources (people, equipment, etc.) are sufficient to cover pretty much the entire target group, and when facilities for clarifying diagnoses, treatment, and follow-up of those with abnormal results have become available. One of the most effective means of treating cancer has been early detection and rigorous application of curative methods. To date, approaches to early detection of cancer have included endoscopic diagnosis, imaging diagnosis, tumor marker diagnosis, endoscopic ultrasonography, and histopathological diagnosis [5]. High tumor marker levels can indicate cancer. Tumor marker testing, when combined with other tests, can assist doctors in detecting and treating specific types of cancer. Tumor marker tests are not optimal. They are not usually specific for cancer, and they may be ineffective at detecting a recurrence. The presence of tumor markers alone cannot be used to diagnose cancer. Other tests are very definitely needed to learn more about a possible malignancy or recurrence. However, these methods also have significant shortcomings: common shortcomings include time-consuming procedures, invasive examination methods (such as for histopathological diagnoses), analytical requirements, and a high need for very specialized training and knowledge that not even all medical professionals might have [6]. Even imaging-based methods of diagnosis are not always able to adequately analyze early examples. While tumor markers used for evaluation are available, they are not always effective and cannot always be identified early enough to provide treatment in a timely manner, thus creating further need for the development of an accurate and rapid method for the early diagnosis of cancer [7]. Moreover, artificial intelligence may be able to identify and diagnose colorectal cancer as well as or better to pathologists by reviewing tissue images. Artificial intelligence might assist pathologists in meeting the growing demand for their services. According to experts, early cancer detection focuses on recognising symptomatic individuals as soon as possible so that they have the highest chance of a successful therapy. When cancer therapy is delayed or unavailable, there is a reduced likelihood of survival, an increase in treatment complications, and an increase in treatment expenses [8, 9]. Cancers are definitely more effectively treated in the early stages, resulting in less physical, mental, and financial misery. Cancer is also one of those medical disorders that has no evident indications or indicators and hence can go unnoticed for a long period within the body [10, 11]. Spatial data from testing can be acquired by utilizing fluorescence hyperspectral imaging (FHSI), which makes it to map out images at the pixel level and makes it possible for researchers to work at capacities that cannot be accomplished utilizing the more customary optical imaging strategies. While these strategies still come with restrictions, there are also promising insights. Machine learning approaches are classified into three types: supervised, unsupervised, and semisupervised. The labelled training data is transferred to the intended output in supervised learning. Unsupervised learning uses unlabelled training data to identify patterns. Using the provided genes, comparable results were obtained. However, only labelled data is used in most cancer prediction studies, whereas large amounts of unlabelled data are excluded. In practice, the label information is usually difficult to get since labelling is expensive, time-consuming, and error-prone. However, the shallow nature of the most commonly used dimension reduction methods outlined above limits the capacity to automatically obtain important high-level information from input data. Deep learning is regarded as a significant achievement in machine learning compared to traditional machine learning methods.

Accurate early prediction is crucial for effective therapy and can enhance cancer outcomes [12]. Scientists employed a variety of methods, including early-stage screening, to discover cancer forms before they developed symptoms. They have also developed new methods for forecasting cancer therapy results in the early stages [13, 14]. Large volumes of cancer data have been collected and made available to the medical research community as a result of the introduction of new medical technology. On the other hand, accurately predicting the fate of an illness is one of the most interesting and difficult undertakings for clinicians [15, 16]. Over the last few decades, similar technologies have seen increased application in a variety of clinical imaging domains, including endoscopy [17], pathology, and CT imaging. Such instruments, for example, can make endoscopic decisions that include the extraction of image highlights, potentially leading to the early detection of malignant growth, the recognition of precancerous conditions, the improvement of amplifying endoscopy with restricted band imaging, and the use or even advancement of Raman endoscopy [18]. These finding methods include the programmed distinguishing proof of malignancy and the discovery of diseases via slide imaging, just as CT conclusions can also zero in on and identify preoperative peritoneal metastasis. As a result, we may argue that computerised reasoning, such as AI, plays an important role in detecting, and hence treating, malignant development that would otherwise result in terminal cancer.

## 2. Background Study

The TNM system is a classification tool used to describe various levels of cancer. Here, T stands for tumor, N stands for node, and M stands for metastasis. Using the TNM system, the “T” plus a letter or number (0 to 4) is used to show how far up or away from its original starting point the tumor has grown, and in the case of cancers, this means how far into the wall of the stomach. The TNM system's numerical classifications are as follows [19–21]:

- Tis: tumor “in situ” that is caught very early and has not grown beyond stomach lining
- T1: tumor has grown through lining and into connective tissue
- T2: tumor has grown into thick inner muscle
- T3: tumor has spread through outer lining but not to any nearby organs or tissues
- T4: tumor has spread into nearby tissues or organs

Meanwhile, the “N” denotes lymph nodes, which are small, bean-shaped organs that assist with combatting disease. The general forecast for patients with malignancy depends on its territorial lymph nodes, which can indicate how far the disease has progressed. The levels of this subsystem are as follows:

- N0: no nodes
- N1: 1 to 6 nodes
- N2: 7 to 15 nodes
- N3: >15 nodes

Finally, the “M” indicates whether the tumor has extended to other parts of the patient's body, in the process also known as differential metastasis. This part of the system only comes in two parts, which are as follows:

- M0: no metastasis
- M1: metastasis

Using these three substages, doctors assign the stage of a patient's cancer by combining the T, N, and M classifications in overall stages [22–24]. The combinations for cancer specifically are outlined here.

- Stage 0 (carcinoma in situ): surgery usually cures this stage, as doctors remove that part of the stomach as well as nearby lymph nodes
- Stage I: in stage IA, cancer spreads into the submucosa (layer next to the mucosa) of the stomach wall, but not yet to any lymph hubs or other organs (T1, N0, and M0). Meanwhile, stage IB signifies that the cancer has grown into the interior levels of the stomach wall and extended to 1 or 2 lymph nodes but not any further (T1, N2, and M0). This IB stage cancer may have also spread into the exterior muscular layers of the stomach wall but not yet to the lymph nodes or other organs (T2, N0, and M0)
- Stage II: surgery to remove that portion of the stomach and/or nearby lymph nodes is still the main treatment, though it is compulsory to receive chemotherapy (“chemo”) or chemo radiation treatments beforehand. In stage IIA, malignant growths expand into the inside layer of the stomach divider and have also spread to between 3 and 6 lymph hubs (T1, N2, and M0). Likewise, cancer in this stage spreads to the outside layers such as the stomach divider, and to 1 to 2 lymph nodes there (T2, N1, and M0), or just to the connective tissue outside the stomach but not the peritoneal coating, serosa, or any lymph nodes (T3, N0, and M0). However, in stage IIB, malignant growths expand into the internal layers and outside solid layers of the stomach divider just as its connective tissue which stretches out either to the peritoneal covering or serosa. This stage may also spread into 7 to 15 lymph nodes (T1, N3a, and M0), 3 to 6 lymph nodes (T2, N2, and M0), 1 to 2 lymph nodes (T3, N1, and M0), or no lymph nodes at all (T4a, N0, and M0)
- Stage III: in stage IIIA, cancer spread deep into the external strong layers of the stomach divider as well as 7 to 15 lymph hubs (T2, N3a, and M0). Moreover, this malignant growth expands into all the levels of the muscle and the stomach's connective tissue, but not the peritoneal coating or serosa. It may also have spread into 3 to 6 lymph nodes (T3, N2, and M0), 1 to 2 lymph nodes (T4a, N1, and M0), or, more rarely, not into any lymph nodes or other organs hubs or far off pieces of the body (T4b, N0, and M0). However, in stage IIIB, cancer has spread into the nearby organs, which may include the spleen, colon, liver, pancreas, kidneys, adrenal organs, or small digestive tract. Here, stage IIIB cancer also expands into the innermost mass of the stomach, the external solid levels of the stomach divider, and at least 16 lymph hubs (T1 or T2, N3b, and M0). Moreover, this cancer grows into the muscular layer and/or the stomach's connective tissue but not to the peritoneal lining or serosa; it may also spread to 7 to 15 lymph nodes (T3, N3a, and M0) or grow into the peritoneal lining or serosa (T4a, N3a, and M0). In other substages, such as T4b, N1 or N2, and M0, the cancer might or might not spread into 1 to 6 lymph nodes excluding different parts of the body. However, in stage IIIC, cancer grows to all muscular layers of the connective tissue found outside the stomach, its peritoneal lining, and its serosa as well as to nearby organs. It may also spread to 16 (T3 or T4a, N3b, and M0), 7, or more lymph instead of other parts of the body (T4b, N3a or N3b, and M0)
- Stage IV: stage IV tumors of any size have spread to different parts of the body as well as surrounding areas of the stomach. Stage 4 cancer is usually referred to as metastatic cancer since it indicates that the illness has spread from its original place to other parts of the body. This stage may be identified years after the initial cancer scare and/or after the primary tumor has been treated

### 2.1. Cancer Diagnosis

Medical experts use various diagnostic tools to search for, detect, and examine threats of cancer, as well as its spread to other parts of the body in metastasis. For example, imaging diagnostics can reveal whether the infection has extended, but there are also a range of other options available for diagnosing risk. The diagnosis techniques [25–28] are listed below.

- Biopsy: this is the expulsion of a limited quantity of cells for assessment under magnification. Depending on a variety of circumstances—including technician experience, skill levels, and equipment—biopsies can result in different, and sometimes inaccurate, diagnoses, and the method is not infallible
- Molecular testing of the tumor: for malignancies, testing might be accomplished for PD-L1 and high microsatellite unsteadiness (MSI-H), which may also be known as a bungle fix lack. Likewise, testing should be able to decide whether the tumor is making an over-the-top protein called human epidermal development factor receptor 2 (HER2), especially if the disease is further developed
- Endoscopy: in this method, medical experts look inside the body with a slim, versatile pipe called a gastro degree. The chamber in patient is implanted through the mouth down the throat as well as in to the stomach and little entrail. The expert can kill tissues and detects its signs of infection
- Endoscopic ultrasound: in some ways, this method resembles the endoscopy previously mentioned. However, it comes with the addition of a little ultrasound test on the end, one whose function is to form an image of internal organs. The stomach divider's ultrasound image is intended to help medical experts assess how far the danger has extended
- Computed tomography (CT) scan: this test utilizes x-rays taken from various points to examine specific internal areas of the body, which are consolidated into a three-dimensional image that shows any variations from the norm, such as tumors. Because of this, a CT sweep can be utilized to gauge the existence, location, and/or size of tumors
- Magnetic resonance imaging (MRI): it is based on the magnetic field that produces relevant pictures of the body and is used to calculate the size of a tumor. Contrast medium, which is a special dye, is provided to the patient before the scan in order to produce a clear image and is also incorporated into the patients' veins
- Positron emission tomography: is normally combined with a CT check and sometimes additionally with a PET-CT filter. A PET output consists of images of cells that are present internally in the body. To obtain these, a limited quantity of a radioactive material is infused into the body. At that point, a scanner can distinguish liquid to deliver internal images of the human body [29]
- Laparoscopy: in this approach, specialist embeds a small cylinder called a laparoscope in to the stomach depression. This device is utilized to see whether the disease has spread to or beyond the coating of the stomach hole or liver [30]. A laparoscope is a modified keyhole surgical endoscope (also known as laparoscopic surgery). Laparoscopic surgery, which requires just a small incision, can be used to perform appendectomies (removal of both the appendix), hysterectomies (removal of both the uterus), and prostatectomies (removal of prostate tissue)
- Blood tests: blood tests that gauge organ capacity can demonstrate whether different organs in the body, for example, the liver, might be influenced by malignant growths such as gastric cancer

### 2.2. Treatments of Cancer

The multiple cancer treatment techniques used to cure cancer are listed below [31–33]:

- Surgery: options may include the removal of the piece of stomach directly influenced by malignant growths during subtotal gastrectomy or removal of the whole stomach during complete gastrectomy. In this situation, the throat is connected straightforwardly to the small digestive system to permit the food to travel through the stomach-related framework, and evacuation of lymph nodes in the midsection is prioritized as needed
- Endoscopic mucosal resection (EMR): EMR is accomplished with the use of a long, thin cylinder loaded with a light, camcorder, and many tools. During EMR of the upper stomach-related area, the cylinder is passed down the patient's throat to arrive at an irregularity in the throat, stomach, or upper piece of the small digestive tract. This particular treatment comes with dangers including narrowing of the throat, cuts, and so forth, even extending to death. Endoscopy has advanced in recent years, allowing a variety of surgeries to be done using a modified endoscope. As a consequence, the procedure is less disruptive. Gallbladder removal, fallopian tube sealing and tying, and excision of small tumors from the gastrointestinal process or lungs are all becoming routine treatments
- Chemo treatment: can be utilized to decimate any disease symptoms that remain after another medical procedure or used to slow the tumor's development or decrease malignant growth-related side effects. The greater part of its use against cancer in particular depends on the specific mix of accompanying medications, which may include cisplatin (accessible as a conventional medication), oxaliplatin (Eloxatin), and/or fluoruracil (5-FU, Efudex). Likewise, the efficacy of these treatments may rely upon the individual being treated and the portion utilized, but as a general rule, chemotherapy can incorporate exhaustion, danger of contamination, queasiness, regurgitating, balding, loss of hunger, and the run
- Radiation therapy: likewise, radiation treatment can be utilized after a medical procedure in order to get rid of any smaller patches of ill tissue or cells that may remain or for particularly malignant growths that cannot be treated with other medical treatments. Radiation therapy (also known as radiotherapy) is a treat symptoms and diseases dose of radiation to eliminate cancer cells and shrink tumors. Radiation is used in x-rays at low doses to see inside your body, such as for teeth or damaged bones. Procedure does not quickly destroy cancer cells. It might take days or weeks of treatment to break the DNA of cancer cells enough to destroy them. Cancer cells continue to die after radiation therapy for weeks or months
- Targeted therapy: a medical specialist may test the malignancy of particular cells to see which focused treatments will work best against them. Directed treatment of malignant growths in the specific region may incorporate specific types
- Immunotherapy: this is a medication therapy that encourages safe frameworks as a means of battling malignant growth. The body's own infection-battling frameworks sometimes do not attach certain diseases on the grounds that the malignant cells produce proteins that make it hard for the resistant framework cells to perceive the disease cells as risky. Immunotherapy and similar treatments work by meddling with that cycle [34]
- Palliative care: consideration experts work with the individual, their family, and their PCPs to provide an additional layer of help that supplements the ongoing care. Palliative consideration can be utilized while going through other more forceful therapies, such as medical procedures, chemo treatment, and radiation treatment. Palliative consideration is provided by a group of specialists, medical attendants, and other exceptionally prepared experts [35]. Palliative consideration groups are meant to improve personal wellbeing and satisfaction for patients and their families, alongside other forms of treatment or healing the individual might be undergoing

## 3. Literature Survey

In 2020, [36] analyzed a neural network (NN) structure validated using 10-fold cross-validation. The neural networks and ensemble learning approach attained higher accurateness as compared to other techniques. Also, the models were validated on a mesothelioma dataset. The greater availability and integration of many data types, such as genomic, transcriptomic, and histopathology data, is allowing cancer therapy to shift toward precision medicine. The use and interpretation of a range of high-dimensional data types requires a significant amount of time and knowledge for translational research or therapeutic operations. Furthermore, merging many data types necessitates more resources than understanding individual data types, as well as modelling algorithms capable of learning from a large number of complex elements [37, 38]. An experimental work [39] in 2021 was carried out on three real datasets (diabetes, heart, and cancer) derived from the UCI repository. This study suggested a neural network-based ensemble learning methodology for the classification of diseases. The computational model achieved appreciable accurateness of 98.5, 99, and 100% on the diabetes dataset, heart dataset, and cancer dataset, respectively. Another recent study [40] in 2021 put forward a CNN algorithm to predict the metastasis status of prostate cancer patients. The classification approach presented favorable outcomes. The mean AUROC achieved by the neural model is 68%. CNNs established their significance classification performance in another latest study [41] carried out in 2021 as well. This study employed CNNs to predict lung cancer. The dataset used in the study was a real-time dataset embracing 311 cancer patients. CNNs were used to derive the important feature, and further, ML models like SVM and KNN was used for the classification of cancer. The classification models performed well and achieved a 71% AUC score. Another efficient hybrid deep learning model was proposed in 2021 [42] to diagnose prostate cancer using histopathological images. A novel image segmentation technique, named RINGS (Rapid IdentificatioN of Glandural Structures), was in this article. This method achieved 90% accurateness and outperformed all the state-of-the-art methods. Firstly, a deep learning technique was employed to extract the regions with higher mitosis activity. Then, SVM model predicted the final tumor proliferation. The projected scheme achieved a 74% accuracy and outperformed all previous approaches significantly [43].

In 2021, a remarkable research [44] was conducted to analyze skin lesion images for skin cancer prediction. The research study conducted an in-depth analysis and identified the major encounters in skin cancer detection. This study also analyzed the performance of the conventional models and proposed the ensemble-based deep learning models for improved prediction performance. Another article in 2021 [45] focused on breast cancer prediction by SEER dataset using ANN approaches. This study disclosed that preprocessing methods can improve the cancer prediction outcomes. In 2021, [46] constructed an ensemble learning model to predict cervical malignancy. The dataset used in the study was derived from the UCI repository. This study used KNN imputations to fill the missing data and also employed data balancing techniques. The dataset was an imbalanced one; hence, data was balanced using the oversampling technique. Random forest feature selection derived the most significant risk factors. The ensemble architecture suggested in the study performed significantly and achieved a 99% AUC score. An *empirical study* was carried out in 2021 [47] which offered a novel classification approach based on ensemble learning. The ensemble algorithm was evaluated on five benchmark datasets from the UCI repository. The model was further compared with 13 classification approaches. The ensemble algorithm achieved an AUC score of 98%, 93%, 99%, 97%, and 99.8% on the cervical cancer dataset, mesothelioma dataset, breast cancer dataset, prostate cancer dataset, and hepatitis C virus, respectively.

## 4. Proposed Architecture

Several strategies for gene selection in cancer categorization have been proposed in prior studies. Deep learning has had a significant impact on a wide range of machine learning applications and research. Technology is crucial for rapidly identifying cancer, and different researchers have presented their findings in a variety of ways. To solve this issue, numerous computer-aided diagnostic (CAD) approaches and systems have been proposed, developed, and implemented. Few of such studies are described in this section. The work flow used for classification of cancer data is shown in Figure 1.

Initially, the exploration of data is done and termed as “exploratory data analysis.” Further, data preprocessing steps are used like cleaning data, reducing dimension (feature reduction), and normalizing the data. Further the preprocessed data in the next stage is divided into training and testing set. The deep learning classification algorithm is trained on the training set for classification of data. The trained classification model is further evaluated on the test set. The evaluation of the data can express the accurateness of the model.

### 4.1. Deep Learning Algorithms

This study proposes to use numerous deep learning algorithms to predict the survivability of colon cancer patient. The research's deep learning methodologies are discussed below.

#### 4.1.1. Artificial Neural Networks

ANN is a method for neural/deep learning inspired by the notion of the human brain. ANN was developed to replicate the functioning of the human brain [48]. The operation of ANNs is somewhat similar to that of biological neural networks. The graphic representation of an ANN is given in Figure 2.

The artificial neural network (ANN) algorithm is only capable of processing numeric and structured data. Perceptrons are single-layer neural networks, whereas ANN comprise of multilayer perceptrons. A neural network may include several layers. Each layer contains one or more neurons or units. Each neuron in the system is linked to every other neuron. Each layer might be assigned a different activation function. Each neuron in layer (*l*) executes the mathematical operation specified in

(1) $$\begin{array}{c} y_{k}^{\left[l\right]}=q_{k}^{t}.a^{\left[l-1\right]}+b_{i}a_{k}^{\left[l\right]}=g^{\left[l\right]}\left(z_{i}^{\left[l\right]}\right). \end{array}$$

The *b*_*i*_ and *t* signify the bias and *activation function*, respectively. The two phases of ANN are forward propagation and reverse propagation. Thus, forward propagation's primary purpose is to multiply weights and add bias, then apply an activation function to the inputs, and propagate it forward. The process of layer updating is given in

(2) $$\begin{array}{c} y_{1}^{\left[2\right]}=q_{1}^{t}.a^{\left[1\right]}+b_{1}a_{1}^{\left[2\right]}=g^{\left[2\right]}\left(z_{1}^{\left[2\right]}\right), \end{array}$$

(3) $$\begin{array}{c} y_{2}^{\left[2\right]}=q_{2}^{t}.t^{\left[1\right]}+b_{2}t_{2}^{\left[2\right]}=g^{\left[2\right]}\left(z_{2}^{\left[2\right]}\right), \end{array}$$

(4) $$\begin{array}{c} y_{3}^{\left[2\right]}=q_{3}^{t}.t^{\left[1\right]}+b_{3}t_{3}^{\left[2\right]}=g^{\left[2\right]}\left(z_{3}^{\left[2\right]}\right), \end{array}$$

(5) $$\begin{array}{c} y_{4}^{\left[2\right]}=q_{4}^{t}.t^{\left[1\right]}+b_{4}t_{4}^{\left[2\right]}=g^{\left[2\right]}\left(z_{4}^{\left[2\right]}\right), \end{array}$$

(6) $$\begin{array}{c} y_{5}^{\left[2\right]}=q_{5}^{t}.t^{\left[1\right]}+b_{5}t_{5}^{\left[2\right]}=g^{\left[2\right]}\left(z_{5}^{\left[2\right]}\right), \end{array}$$

(7) $$\begin{array}{c} y_{6}^{\left[2\right]}=q_{6}^{t}.t^{\left[1\right]}+b_{6}t_{6}^{\left[2\right]}=g^{\left[2\right]}\left(z_{6}^{\left[2\right]}\right). \end{array}$$

By modifying the activation functions of the output layers, ANNs may be employed for regression and classification problem. The sigmoid activation function used for construction of CNN is given in

(8) $$\begin{array}{c} g\left(y\right)=\frac{1}{1+e^{-y}}. \end{array}$$

The most critical stage is backpropagation, which involves identifying the model's optimum parameters via backpropagating the neural network layers. Backpropagation requires an optimization function to determine the optimal weights for the model.

#### 4.1.2. Convolutional Neural Networks (CNN)

A CNN is distinct from a standard neural network in that it operates over a large number of inputs. Each layer searches for patterns or uses data included within the data [49]. Convolutional neural networks (CNNs), a form of artificial neural network prominent in computer vision, are finding traction in a variety of sectors, including radiology. CNN employs various building elements, including convolution layers, pooling layers, and fully connected layers, to learn geographical information hierarchies instantly and adaptively via backpropagation. The basic CNN architecture is depicted in Figure 3.

Each Conv layer comprises several planes, which enables the generation of multiple feature maps at every location using

(9) $$\begin{array}{c} L\left[m,n\right]=\left(a*b\right)\left[m,n\right]=\underset{i}{\sum }\underset{j}{\sum }b\left[i,j\right]a\left[m-i,n-j\right], \end{array}$$

where *a* and *b* denote the input and [*m*, *n*] is the [row, column] index of the resultant matrix.

We used the CONV1D model to predict cancer patient survival. The model is optimized using the root mean square propagation algorithm. A CNN receives text in the form of a sequence. The embedding layer takes as an input the embedding matrix. Each remark is exposed to a combination of five different filter sizes and GlobalMaxPooling1D layers. After that, all outputs are pooled.

#### 4.1.3. Restriction Boltzmann Machine (RBM)

The Boltzmann machine is a technique for unsupervised modelling. This technique employs probability-based prediction [50].  Figure 4 depicts the structure of a restricted Boltzmann machine.

RBM is a probabilistic, generative technique that is undirected. Since RBM comprises an input layer and a hidden layer, it is also an asymmetrical bipartite graph. Each visible node is associated with each hidden node. This approach was aimed at determining the joint probability distribution that maximizes the logarithmic-likelihood function. The probability distribution is specified in

(10) $$\begin{array}{c} C\left(v_{i}=1\;|\;Y\right)=\frac{1}{1+e^{-x}}\left(\underset{j}{\sum }w_{ij}Y_{J}+p_{i}\right), \end{array}$$

(11) $$\begin{array}{c} D\left(Y_{i}=1\;|\;Y\right)=\frac{1}{1+e^{-x}}\left(\underset{i}{\sum }w_{ij}v_{i}+q_{j}\right). \end{array}$$

*C* and *D* represent the vectors for the layers with no intralayer connection. Due to the undirected nature of RBMs, the weights are changed through a process called contrastive divergence. At the first step, the weight distribution for input layer nodes is produced arbitrarily and used for the nodes in the hidden layer.

Additionally, the hidden layer's nodes reproduce visible nodes by applying the same weights. Due to their isolation, the formed nodes are not identical. An RBM contains an asymmetric bipartite graph devoid of links between units belonging to the same group.

#### 4.1.4. Autoencoders with a Deep Learning Algorithm

The autoencoder architecture is designed to provide encoding and decoding. Autoencoders function in a compression and decompression fashion [51].  Figure 5 illustrates the construction of a deep autoencoder, which includes the input, hidden, and output layers.

The encoder uses the concept of dimensionality reduction. The loss is calculated using the function “binary cross-entropy.” Equation (12) is used to calculate the cross-entropy (CE).

(12) $$\begin{array}{c} \text{CE}=\frac{1}{j}\overset{j}{\underset{i=1}{\sum }}P_{i}\log\left(L_{i}\right)+\left(1-P_{i}\right)\left(\log\left(1-L_{i}\right)\right). \end{array}$$

The word *L*_*i*_ reflects the probability associated with the *i*^th^ instance, and *P*_*i*_ represents all of the truth values associated with the *j*^th^ occurrence. The activation function employed in deep autoencoders, namely, “RELU,” is presented in

(13) $$\begin{array}{c} f\left(y\right)=\max\left(0,y\right). \end{array}$$

*y* is the input in this case. Additionally, we optimized the method using the “root mean square propagation” optimizer. The root mean square error (RMSE) is determined using

(14) $$\begin{array}{c} \text{RMSE}=\sqrt{\overset{n}{\underset{i=1}{\sum }}\frac{{\left(\alpha_{i}-\beta_{i}\right)}^{2}}{n}}\;, \end{array}$$

where *α*_1_, *α*_2_, *α*_3_, ⋯*α*_*n*_ are the predicted values, *β*_1_, *β*_2_, *β*_3_, ⋯*β*_*n*_ are the observed values, and *n* denotes the number of observations.

The downside of this strategy is that compressed data cannot be organized in its compressed form. To be clear, the encoder does not remove any constraints.

## 5. Results

The prediction outcomes achieved by different learning approaches are presented below in this section. Multiple parameters have been used to assess the performance of ANN, CNN, Deep AE, RBM.

### 5.1. Model Evaluation on Basis of Accuracy

The accuracy scores attained by models are depicted in Figure 6.

The results shown in Figure 6 depict that all the neural learning approaches have shown great performance; the best accuracy score is obtained by deep autoencoder model.

### 5.2. Model Evaluation on the Basis of AUC Scores

The AUC scores attained by models are depicted in Figure 7.

As per Figure 7, deep autoencoder model has attained the highest AUC score (0.95) followed by RBM.

### 5.3. Model Evaluation on the Basis of F1-Score

The F1-scores accomplished by deep learning approaches are depicted in Figure 8.

The highest F1-score is attained by RBM model and the lowest F1-score is attained by artificial neural networks.

### 5.4. Model Evaluation on the Basis of Recall

Figure 9 illustrates the sensitivity (recall) scores attained by deep learning algorithms. The highest recall score is achieved using deep AE and lowest score is attained by CNN.

From Figures 6, 7, 8, and 9, it is clear that these methods have shown great success in detection of early cancer. One can say that deep learning technologies play an important role in detecting, and hence treating, malignant development that would otherwise result in terminal cancer. Deep learning, unlike typical machine learning methods, can detect intricate patterns underneath data and give critical evidence. The performance of different deep learning models is extensively studied to determine which method outperforms the others, and then, the network's prediction accuracy is investigated.

## 6. Discussion

Experiment results show that deep learning-based models perform quiet well. Practically, there exists small amount of labelled data. The little labelled data may not provide enough information to forecast models. Assume we can include high-dimensional data, allowing for the discovery of critical and essential information while avoiding duplication. As a result, the following categorization approach produces more accurate and efficient results.

Multiple deep learning approaches were used to compare the proposed strategy. AEs have identical network topologies as stacked sparse autoencoders except for the lack of a pretraining phase and the sparse restriction.  Section 5 provides the simulation results and reveals that AEs outperform the other three models in terms of accuracy, AUC, and recall scores. In terms of F1-score, RBM displayed the best results followed by autoencoders. This is because these two deep learning algorithms have deep architectures. Unlike traditional machine learning methodologies, deep learning can automatically identify complex patterns beneath data and provide crucial evidence that may be acquired, and discriminative qualities might be studied. Prediction performance is improved by both the recovered information and the underlying structure of the data.

Furthermore, we discover that the AE model beats the other prediction models. The global fine-tuning procedure then optimizes and specifies the entire model's parameters, making classification prediction easier. Furthermore, AEs learn more abstract and representational properties rather than just reconstructing the inputs, making them more successful than AEs for high-dimensional data and categorization. The simulation results show that automated prediction models can accurately estimate the survival of colon cancer patients. Deep autoencoders had the best performance, with a 97 percent accuracy and a 95 percent AUC-ROC (area under curve-receiver operating characteristic). As a result, we might conclude that computerised thinking, such as AI, plays a critical role in recognising and so treating malignant growth that would otherwise lead to fatal cancer.

## 7. Conclusion

Colon cancer is a type of cancer that begins in the large intestine. Cancer prediction and diagnosis is a complicated issue that has aroused international attention due to the disease's high morbidity and fatality rates. Early accurate prognosis is critical for successful treatment and can improve cancer outcomes. Early identification and strict implementation of curative procedures have been two of the most successful approaches to treating cancer. Also, predicting the outcomes of treatments post cancer like therapies (chemotherapy, immunotherapy, and other related therapies) is very important for estimating the survivability of cancer patients. In this study, we evaluated colon cancer data from the SEER programme to generate reliable colon cancer survival prediction models. We compared several categorization methods to determine the risk of death five years following diagnosis. Our study discovered that the deep autoencoder model provided the most significant prediction performance in terms of accuracy and area under the receiver operating characteristic curve. According to the study, detecting and controlling cancer immunotherapy toxicities will be a critical component of treatment efficacy in the future. Personalised combination therapies that employ novel ways to address each patient's disease biology will be the most promising cancer therapy strategies.

## Figures and Tables

**Figure 1:** Deep learning for cancer classification.

**Figure 2:** Artificial neural network (ANN) basic architecture.

**Figure 3:** Framework for CNN.

**Figure 4:** Model representation of RBM.

**Figure 5:** Deep autoencoders.

**Figure 6:** Accuracy scores.

**Figure 7:** AUC scores.

**Figure 8:** F1-score.

**Figure 9:** Recall score.

## Data Availability

Data are available from the corresponding author upon request.
